# Antiviral Therapy for Prevention of Perinatal Hepatitis B Virus Transmission Reduces the Incidence of Postpartum Hepatitis Flare

**DOI:** 10.1155/2022/7046955

**Published:** 2022-07-11

**Authors:** Min Quan, Xiao-Min Liu, Cong Liu, Wei Li, Hui-Chun Xing

**Affiliations:** ^1^Center of Liver Diseases Division 3, Beijing Ditan Hospital, Capital Medical University, Beijing 100015, China; ^2^Peking University Ditan Teaching Hospital, Beijing 100015, China; ^3^Department of Internal Medicine Oncology, Beijing Ditan Hospital, Capital Medical University, Beijing 100015, China; ^4^Department of Infectious Diseases, The Second Hospital of Shanxi Medical University, Taiyuan, Shanxi 030000, China

## Abstract

*Background*: Currently, there are few studies on the effect of prophylactic anti-hepatitis B virus (HBV) therapy (AVT) for mother-to-child transmission during pregnancy on postpartum hepatitis flare (PHF) and the risk factors for postpartum hepatitis flare in women with chronic hepatitis B infection. *Aim*: To analyze the effect of AVT on the postpartum hepatitis flare and risk factors related to postpartum hepatitis flare. *Methods*: This study retrospectively enrolled hepatitis B surface antigen (HBsAg)-positive and hepatitis B e antigen (HBeAg)-positive women with HBV DNA ≥ 10^6^  IU/mL. Six hundred fourteen pregnant women were included: 444 in the anti-HBV therapy group (T-G) and 170 in the control group (C-G). To analyze the risk factors, women with alanine aminotransferase (ALT) flare (ALT > 40 U/L) were assigned to the PHF group (PHF-G, *n* = 355), and all the others were assigned to a non-PHF group (NPHF-G, *n* = 259). *Results*: At 6 weeks postpartum, ALT and AST levels were higher, and ALB levels were lower in the C-G than those in T-G (*P* < 0.05). Also, ALT (at baseline, pregnancy 32nd and 36th, intrapartum), AST (at pregnancy 32nd and 36th week, and intrapartum), HBcAb (at baseline, intrapartum), and HBV DNA (at intrapartum) of PHF-G were significantly higher than those of NPHF-G (*P* < 0.05). Multivariate analysis showed that ALT (OR = 1.067, *P* < 0.001) and HBcAb (OR = 1.213, *P* ≤ 0.001) in pregnant women were risk factors for PHF. The prophylactic anti-HBV for the prevention of perinatal HBV transmission (OR = 0.357, *P* < 0.001) was the protective factor for PHF. *Conclusion*: Pregnant women with prophylactic anti-HBV during the third trimester of pregnancy had a lower incidence of postpartum hepatitis flare, especially a lower risk of serious hepatitis flare. ALT and HBcAb in pregnant women were risk factors for PHF. Women infected with HBV should be closely monitored ALT during pregnancy and postpartum.

## 1. Introduction

Chronic viral hepatitis B is one of the main causes of liver cirrhosis and liver cancer. The positive rate of HBsAg in pregnant women in China is about 6-8%. Infantile infection of HBV is the main cause of chronic hepatitis B, and mother-to-child transmission (MTCT) is the main way of infantile infection with hepatitis B virus [1]. After acute exposure, the risk of developing chronic HBV infection ranges from 90% in newborns of HBeAg- positive mothers to 25% to 30% in infants [2]. Although the use of neonatal immunoglobulin and hepatitis B vaccine reduced the incidence of mother-to-child transmission, mothers with high viral load have been reported to be more likely to transmit HBV to their infants compared to those with low viral load. Prophylactic anti-HBV therapy in the third trimester of pregnancy significantly reduced the incidence of mother-to-child transmission of HBV in mothers with high viremia [3, 4]. However, postpartum hepatitis flared in 25%-44.7% HBV-infected women [5–7]. The existing studies have shown that some of the identified reasons for postpartum hepatitis flare still cannot explain the correlation with HBV. It also remains unclear whether the prophylactic anti-HBV therapy against HBV can reduce the risk of postpartum hepatitis flare. This study evaluated whether prophylactic anti-HBV therapy in the third trimester of pregnancy could reduce the incidence of postpartum hepatitis flare and the effect of anti-HBV therapy on the severity of postpartum hepatitis flare.

The factors that cause postpartum hepatitis flare are complicated. It is well known that some hormones in pregnant women go through immune changes during pregnancy. For example, the increase of adrenocortical hormone, estrogen, and progesterone may have an immunosuppressive effect, and the immune system tends to recover after delivery quickly [8, 9]. It is unknown if immune changes in pregnancy and postpartum impact the natural history of chronic hepatitis B. Higher rates of HBeAg loss (and HBsAg clearance) and biochemical-hepatic flares with increased ALT levels have been reported, especially during early postpartum when immune reconstitution occurs [9]. In the present study, we hoped to find a correlation between postpartum hepatitis flare and hepatitis B virus so as to provide valid references for anti-HBV activity in postpartum hepatitis flare. The correlation analysis between prenatal biochemical screening and postpartum hepatitis flare can provide a preventive basis for predicting postpartum severe hepatitis flare.

## 2. Methods

Pregnant women with serum HBsAg-positive and a high HBV viral load (≥10^6^ IU/mL) were recruited from a single-center of Beijing Ditan hospital, Capital Medical University (in China) between January 2014 and September 2017 so as to observe the effect of AVT for prevention of MTCT on the postpartum hepatitis flare. Pregnant women were assigned into the T-G (444/614) [prophylactic anti-HBV therapy group, treated with lamivudine (LAM) 100 mg/day or telbivudine (LdT) 600 mg/day or tenofovir (TDF) 300 mg/day, during 24th to 29th weeks of pregnancy) or C-G (170/614) (control group, no prophylactic anti-HBV therapy during pregnancy). All prophylactic anti-HBV therapy was discontinued within postpartum 6 weeks. Six hundred fourteen women were also assigned to the postpartum hepatitis flare group (PHF-G) (355/614) or non-PHF-group (NPHF-G, 259/614) based on whether or not they developed PHF. PHF was defined as ALT rise to the upper limit of normal (ULN) during 6 weeks postpartum, with ULN taken as 40 U/L (i.e.,>40 U/L).

Pregnant women were screened for the following eligibility criteria: (i) seropositive for both HBsAg and HBeAg, HBV DNA levels ≥10^6^ IU/ml, ALT, and AST < ULN (40 U/L). The patients with any of the following conditions were excluded: (i) coinfection with hepatitis C, D, or E or human immunodeficiency virus (HIV); (ii) evidence of hepatocellular carcinoma, cirrhosis, or any other disease that could influence the study results; and (iii) concurrent therapy with immune modulators, cytotoxic drugs, or steroids.

Serum levels of HBV DNA, HBsAg, HBsAb, HBeAg, HBeAb, liver function tests, and hematology were measured at 28 (as baseline), 32, and 36 weeks of pregnancy and at 6 weeks postpartum. HBV DNA levels were determined using COBAS AmpliPrep/COBAS Taqman HBV test version 2.0 (Roche Diagnostics). HBV serology was determined using Abbott i2000 reagent.

This research was approved by the Ethics Committee of the Beijing Ditan Hospital, Capital Medical University (jinglundizi 2016-024 No. 01). Written and informed consent was obtained from all participants.

### 2.1. Statistical Analysis

Normally distributed continuous variables were expressed as mean ± standard deviation. Non-normally distributed quantitative data were presented as median and range. The Chi-square test, Fisher's exact test, and ANOVA were used for comparison between the groups using the software IBM SPSS Statistics for Windows, version 19.0 (IBM Corp., Armonk, NY, USA). Clinical correlates were assessed by multivariate analysis using forward stepwise regression. A *P* value < 0.05 was considered as statistical significance.

## 3. Results

### 3.1. Baseline Characteristics

A total of 614 pregnant women met the inclusion criteria. The subject selection process is shown in Figure 1. Baseline demographic and clinical characteristics are shown in Table 1. Pregnant women in the two groups (T-G 444/614, C-G 170/614) had comparable age, parity, HBV DNA, HBeAg, HBeAb, HGB, PLT, ALT, AST, TBIL, DBIL, and ALB (*P* > 0.05), but WBC levels were higher in the T-G (*P* = 0.030). However, the difference in WBC levels was not statistically significant for clinical use.

### 3.2. Effects of AVT for Preventing MTCT during the Third Trimester of Gestation on Postpartum Hepatitis Flare

During 6 weeks of postpartum, the C-G had higher levels of ALT [63.00 (36.55, 158.08) U/L] compared to the T-G [43.00 (26.65, 76.38) U/L] (*P* < 0.001); the same tendency was observed for AST [39.75 (26.98, 92.60) U/L vs. 34.45 (23.73, 53.83) U/L] (*P* = 0.001). The C-G had lower level of ALB [45.70 (44.30, 47.20) vs. 46.20 (44.50, 47.70) g/L]. There were no significant differences in TBIL and DBIL between the two groups (Table 2).

HBV DNA and HBeAg in the T-G group significantly decreased during intrapartum compared to the C-G (*P* < 0.001). The incidence of PHF was (120/170, 70.59%) in the C-G group and (239/444, 52.9%) in the T-G group (Table 3) (*x*^2^ = 15.721, *P* < 0.001). ALT and AST were graded according to different multiples of ULN. The results showed the incidence of ALT or AST exceeding 2 times ULN levels in T-G group which significantly lower than that in C-G group (Table 3). PHF occurs at the highest rate in the patients with 1-2 times ULN of ALT (*n* = 173, 28%) or 1-2 times ULN of AST (*n* = 181, 29.48%) at postpartum 6 weeks, followed by in the patients with 2-5 times ULN of ALT (124, 20%) or 2-5 times of ULN AST(88,14.33%) (*P* ≤ 0.001) (Figure 2, Table 3).

### 3.3. Postpartum Hepatitis Flare Characteristics

Out of a total of 614 subjects, 355 experienced ALT elevation (ALT > 40 U/L) during 6 weeks postpartum. This meant that at least 57.8% (355/614) women infected with HBV had PHF. There was no difference in the incidence of PHF among different parity (*x*^2^ = 3.373, *P* = 0.066). At baseline, there were no significant differences in AST, DBIL, HBeAg, ALB, WBC, HGB, PLT, and HBV-DNA levels between PHF-G and NPHF-G, but there were significant different in ALT, TBIL, and HBcAb levels (*P* < 0.05). However, at intrapartum, HBV DNA load in the PHF-G was significantly higher than that in the NPHF-G (z = −3.102, *P* = 0.002). ALT and AST in the third trimester of gestation were definitely correlated with the incidence of postpartum PHF. The ALT (at baseline, pregnancy 32 and 36 weeks, and intrapartum, respectively), AST (at pregnancy 32 and 36 weeks, and intrapartum, respectively), HBcAb (at baseline and intrapartum, respectively), and HBV DNA (at intrapartum) were significantly higher in PHF-G than in NPHF-G (all *P* < 0.05) (Table 4).

### 3.4. Risk Factors of Postpartum Hepatitis Flare

Multivariate logistic regression analysis showed that ALT (OR = 1.067, *P* < 0.001) at 32 weeks of pregnancy and HBcAb at intrapartum (OR = 1.213, *P* ≤ 0.001) were risk factors for PHF. The prophylactic anti-HBV therapy during the third trimester (OR = 0.357, *P* < 0.001) was a protective factor for PHF (Table 5). It also indicated that prophylactic anti-HBV therapy was effective for preventing postpartum hepatitis flare.

## 4. Discussion

The prevention of HBV perinatal transmission, which is considered to mainly occur at intrapartum, HBIG, and vaccine failures, occurs almost exclusively in pregnant HBeAg-positive women with high HBV DNA levels (200,000 IU/ml and/or HBsAg level above 4–4.5 log10 IU/ml) [6, 10–12]. At present, global guidelines recommend that pregnant women infected with HBV with high viral load (>6 log copies or >200,000 IU/mL) [13–15] in the third trimester should be given anti-HBV therapy to prevent the risk of mother-to-child transmission of hepatitis B virus [11]. A large number of studies have shown that prophylactic anti-HBV therapy in the third-trimester pregnancy can effectively reduce HBV DNA viral load, showing the clear effect of preventing infection in infants [10, 14, 16–19], and no increased risk of an infant or maternal safety outcomes after prophylactic anti-HBV therapy [20]. The probability of postpartum hepatitis flare in pregnant women with a high viral load of HBV is significantly higher than that in non-HBV infected women [21]. However, few studies have addressed the effect of prophylactic anti-HBV therapy on postpartum hepatitis flare. Several studies have indicated that women taking anti-HBV therapy during the third-trimester pregnancy had significantly higher postpartum hepatitis flare after delivery than those without prophylactic anti-HBV therapy [6, 22]. Other research showed that anti-HBV therapy could not reduce the incidence of postpartum hepatitis flare [8], which was inconsistent with our results. We found that the risk of postpartum hepatitis flare in the prophylactic anti-HBV therapy group was significantly lower than the non-anti-HBV therapy group of pregnant women with high viral load, especially in the relatively severe hepatitis flare women with ALT >5ULN (>200 U/L). It also indirectly reflects that part of the postpartum hepatitis flare is related to HBV. Therefore, we speculated that these postpartum women may benefit from postpartum anti-HBV therapy but needs to be examined over the longer follow-up time.

The immune status of pregnant women with chronic HBV infection is different from that of chronic HBV-infected women who are not pregnant [23]. Rapid changes in postpartum immune status and the resulting rebound of the inflammatory response may lead to postpartum hepatitis flare [24]. Due to the unique immune changes during pregnancy, 25% of women with chronic hepatitis B demonstrate increased liver inflammation in the postpartum period [5, 25]. Others reported that hepatitis flared in 25%–44.7% of untreated women [5–7] and was more likely to occur in HBeAg-positive women [5]. The results of our study showed that the postpartum hepatitis flare rate in HBV pregnant women with high viral load (median7.75) was 58% and the incidence of PHF was higher than that previously reported, which may be due to the fact that there was no HBeAg-negative hepatitis B infection in the women included in this study. Previous studies showed that the incidence of PHF in HBeAg-positive patients was significantly higher than that in HBeAg-negative patients [5]. The characteristics of T cell immunity differed between mothers with postpartum hepatitis flare and those without hepatitis flare from pregnancy to postpartum. The results indicated that maternal immune status might have an important role in postpartum hepatitis flare in HBV-infected mothers [23]. It has been suggested that pregnancy period may be the break of immune tolerance and the best period for anti-HBV therapy [26]. Further studies of the immunopathogenesis of pregnancy-related flare, as well as effects on long-term outcomes of the mother to guide anti-HBV therapy during postpartum hepatitis flare, are needed.

As for the risk factors of PHF, it is of great importance to predict the occurrence of PHF. However, there are only a few relevant studies [27]. One retrospective cohort study of 38 pregnancies demonstrated a high rate of postpartum liver flare (45%), but they did not provide any information that could clearly predict PHF [24, 27]. Our retrospective study showed that women with elevated ALT or HBcAb during pregnancy were prone to PHF, which was similar to the study of Liu et al. [7]. All the results suggested that patients most likely to develop PHF were those with HBeAg-positive, high levels of HBcAb, and ALT. Therefore, these women should be followed-up more closely.

This retrospective study has a few limitations. First, the therapy assignment was not performed by randomization. Second, given that the postpartum bloods were taken between 6 weeks and 9 weeks after delivery, there is the possibility that flares occurring very early (<4 weeks) or late (>9 weeks) would have been missed.

## 5. Conclusion

The proportion of pregnant women with high viral load and HBsAg-positive with postpartum hepatitis flare is not low, which is worth paying attention to. Prophylactic anti-HBV therapy during pregnancy could reduce the risk of mother-to-child transmission and reduce the incidence of postpartum hepatitis flare and the risk of severe hepatitis flare. Long-term follow-up studies are needed to determine the clinical benefits of prolonged anti-HBV therapy following the special period of puerperal immune fluctuations.

## Figures and Tables

**Figure 1:** Summary of analytic sample, and antiviral treatment (PHF, postpartum hepatitis flare).

**Figure 2:** (a) Comparison of proportion of postpartum ALT level (classification based on multiples of ULN) in anti-HBV therapy group (T-G) vs. no anti-HBV therapy group (C-G). (b) Comparison of proportion of postpartum AST level in T-G vs. C-G.

**Table 1:** Baseline characteristics of T-G and C-G.

Baseline characteristics	Group 1:C-G (*n* = 170)	Group 2:T-G (*n* = 444)	t/Z/x^2^	*P*
	M (P25, P75)	M (P25, P75)		
Age (years)	28 (26, 30)	29 (26, 31)	−1.553	0.120
WBC (×10^9^/L)	8.67 (7.35, 10.21)	9.01 (7.76, 10.42)	−2.172	0.030
HGB (g/L)	118 (110.75, 125.00)	119 (111.00, 124.00)	−0.712	0.476
PLT (×10^9^/L)	193.50 (162.75, 228.00)	195.50 (167.75, 227.00)	−0.440	0.660
ALT (U/L)	17.95 (14.50, 22.80)	17.80 (14.10, 23.88)	−0.215	0.830
AST (U/L)	18.30 (15.88, 21.43)	18.50 (15.80, 22.35)	−0.217	0.828
TBIL (umol/L)	7.00 (5.50, 7.90)	6.65 (5.62, 8.28)	−0.651	0.515
DBIL (umol/L)	1.40 (1.10, 1.80)	1.40 (1.10, 1.80)	−0.493	0.622
ALB (g/L)	37.30 (35.80, 38.80)	37.35 (35.80, 38.88)	−0.022	0.983
HBeAg(S/CO)	1339.58 (1313.27, 1539.86)	1339.58 (1316.00, 1519.73)	−0.374	0.708
HBcAb(S/CO)	10.19 (9.87, 11.14)	10.19 (9.71, 10.98)	−0.591	0.554
HBV-DNA (log_10_IU/mL)	7.78 (7.19, 8.23)	7.88 (7.46, 8.23)	−1.539	0.124
Start antiviral time (pregnant weeks)		28(26, 28)		
Parity				
Primiparity	*n* = 95 (55.9%)	*n* = 270 (60.8%)	1.239	0.266
Multiparity	*n* = 75 (44.1%)	*n* = 174 (39.2%)		
Type of anti-viral therapy				
Lamivudine		*n* = 39 (6.3%)		
Telbivudine		*n* = 397 (64.6%)		
Tenofovir		*n* = 8 (1.3%)		

ALT: alanine aminotransferase; AST: aspartate aminotransferase; TBil: total bilirubin; DBIL: direct bilirubin; HBeAg: hepatitis B e antigen; HBsAg: hepatitis B surface antigen; HBV: hepatitis B virus; HBV DNA: hepatitis B deoxyribonucleic acid; SD: standard deviation; ULN: upper limit of normal; WBC: white blood cell; PLT: platelet; HGB: hemoglobin; ALB: albumin; T-G: anti-HBV therapy group; C-G: no anti-HBV therapy group.

**Table 2:** Comparison of postpartum liver function in C-G versus T-G.

	C-G M (P25, P75)	T-G M (P25, P75)	Z	*P*
Postpartum 6 w				
ALT (U/L)	63.00 (36.55, 158.08)	43.00 (26.65, 76.38)	−5.312	<0.001
AST (U/L)	39.75 (26.98, 92.60)	34.45 (23.73, 53.83)	−3.431	0.001
TBIL(umol/L)	10.45 (8.28, 13.08)	10.50 (8.53, 13.08)	−0.626	0.532
DBIL(umol/L)	2.85 (2.30, 3.80)	3.00 (2.30, 3.90)	−1.235	0.217
ALB(g/L)	45.70 (44.30, 47.20)	46.20 (44.50, 47.70)	−2.453	0.014
Intrapartum				
ALT (U/L)	16.10 (12.65, 21.20)	16.5 (12.60, 23.60)	−1.007	0.314
AST (U/L)	19.1 (16.60, 22.65)	20.90 (16.80, 26.40)	−2.854	0.004
TBIL (umol/L)	7.30 (6.30, 8.90)	7.40 (6.10, 9.10)	−0.051	0.959
DBIL (umol/L)	1.60 (1.20, 1.95)	1.60 (1.20, 2.20)	−0.756	0.045
ALB (g/L)	35.70 (33.45, 38.00)	35.90 (33.50, 37.60)	−0.043	0.965
HBeAg (S/CO)	1465.76 (1246.30, 1604.95)	1312.40 (1077.22, 1463.02)	−4551	<0.001
HBcAb (S/CO)	10.08 (8.76, 10.86)	9.78 (8,51, 10.91)	−0.857	0.391
HBV-DNA (log10 IU/mL)	7.81 (7.27, 8.23)	3.93 (3.31, 4.56)	−18.09	<0.001

ALT: alanine aminotransferase; AST: aspartate aminotransferase; TBil: total bilirubin; DBIL: direct bilirubin; ALB: albumin; HBeAg: hepatitis B e antigen; HBsAg: hepatitis B surface antigen; HBV: hepatitis B virus; HBV DNA: hepatitis B deoxyribonucleic acid; T-G: anti-HBV therapy group; C-G: no anti-HBV therapy group.

**Table 3:** Characteristics of different degrees of PHF.

Postpartum 6 w		C-G (*n*)	(*n*/170)	T-G (*n*)	(*n*/444)	*z*	*P*	Overall (*n*)	(*n*/614)
ALT						*z* = −5.416	<0.001		
≤1 × ULN	≤40	50	29.40%	209	47.10%			259.00	42.18%
>1 × ULN	>40	120	70.59%	235	52.93%			355.00	57.82%
1-2 × ULN	41-80	44	25.88%	129	29.05%			173.00	28.18%
2-5 × ULN	81-200	43	25.29%	81	18.24%			124.00	20.20%
5-10 × ULN	201-400	26	15.29%	22	4.95%			48.00	7.82%
≥ 10 × ULN	≥401	7	4.12%	3	0.68%			10.00	1.63%
AST						*z* = −3.249	0.001		
≤1 × ULN	≤35	75	44.12%	231	52.03%			306.00	49.84%
>1 × ULN	>35	95	55.88%	213	47.97%			308.00	50.16%
1-2 × ULN	35-70	39	22.94%	142	31.98%			181.00	29.48%
2-5 × ULN	70-175	34	20.00%	54	12.16%			88.00	14.33%
5-10 × ULN	175-350	18	10.59%	14	3.15%			32.00	5.21%
≥ 10 × ULN	≥350	4	2.35%	3	0.68%			7.00	1.14%

ALT, alanine aminotransferase; AST,aspartate aminotransferase; ULN, upper limit of normal; T-G, anti-HBV therapy group, C-G, no anti-HBV therapy group.

**Table 4:** Comparison between PHF-G and NPHF-G.

Baseline characteristics	NPHF-G (*n* = 259)	PHF-G (*n* = 355)	t/Z/x^2^	*P*
	n/%, M (P25, P75)	*n*/%, M (P25, P75)		
Age (years)	28.00 (26.00, 31.00)	29.00 (26.00, 31.00)	z = −1.793	0.073
≦30	192 (74.1%)	240 (67.6%)	x^2^ = 3.058	0.080
>30	67 (25.9%)	115 (32.4%)		
WBC (×10^9^/L)	9.01 (7.44, 10.42)	8.83 (7.68, 10.28)	z = −0.008	0.994
HGB (g/L)	119.00 (110.00, 125.00)	118.00 (111.00, 124.00)	z = −0.126	0.900
PLT (×10^9^/L)	197.00 (167.00, 236.00)	191.50 (164.00, 225.00)	z = −1.242	0.214
ALT (U/L) baseline	17.10 (13.70, 22.00)	18.60 (14.80, 24.75)	z = −3.384	0.001
ALT (U/L) 32 w	14.05 (10.80, 17.55)	17.40 (13.70, 25.60)	z = −7.424	<0.001
ALT (U/L) 36 w	15.10 (12.08, 19.00)	17.05 (13.50, 23.40)	z = −5.247	<0.001
ALT (U/L) intrapartum	14.20 (11.10, 18.60)	17.90 (13.60, 26.70)	z = −6.719	<0.001
AST (U/L) baseline	18.10 (15.40, 21.7)	18.60 (16.05, 22.50)	z = −1.201	0.230
AST (U/L) 32 w	18.10 (15.45, 21.90)	20.05 (17.13, 26.28)	z = −5.022	<0.001
AST (U/L) 36 w	17.60 (15.00, 20.70)	18.80 (16.10, 22.20)	z = −3.366	0.001
AST (U/L) intrapartum	18.80 (15.28, 22.45)	21.30 (17.80, 27.83)	z = −5.572	<0.001
TBIL (umol/L)	7.00 (5.80, 8.80)	6.50 (5.50, 7.80)	z = −3.070	0.002
DBIL (umol/L)	1.50 (1.10, 1.80)	1.30 (1.10, 1.70)	z = −1.514	0.130
ALB (g/L)	37.30 (35.80, 38.60)	37.30 (35.70, 39.00)	z = −0.211	0.833
HBeAg (S/CO)	1406.02 (1263.21, 1560.89)	1421.18 (1220.19, 1600.57)	z = −0.380	0.704
HBcAb (S/CO) baseline	10.08 (8.31, 11.25)	10.67 (9.64, 11.63)	z = −4.015	<0.001
HBcAb (S/CO intrapartum	9.22 (7.45, 10.37)	10.21 (9.21, 11.04)	z = −6.411	0.000
HBV-DNA (log_10_IU/mL) baseline	7.89 (7.50, 8.23)	7.84 (7.35, 8.23)	z = −1.083	0.279
HBV-DNA (log_10_IU/mL) intrapartum	4.21 (3.46, 5.18)	4 (3.68, 7.34)	z = −3.102	0.002
Parity				
Primiparity	165 (63.7%)	200 (56.3%)	x^2^ = 3.373	0.066
Multiparity	94 (36.3%)	155 (43.7%)		
Anti-viral therapy				
No	50 (19.3%)	120 (33.8%)	x^2^ = 15.721	<0.001
Yes	209 (80.7%)	235 (66.2%)		
Type of anti-viral therapy				
Lamivudine	24	15		
Telbivudine	180	217		
Tenofovir	5	3		

ALT: alanine aminotransferase; AST: aspartate aminotransferase; TBil: total bilirubin; DBIL: direct bilirubin; HBeAg: hepatitis B e antigen; HBsAg: hepatitis B surface antigen; HBV: hepatitis B virus; HBV DNA: hepatitis B deoxyribonucleic acid; SD: standard deviation; ULN: upper limit of normal; WBC: white blood cell; PLT: platelet; HGB: hemoglobin; ALB: albumin; PHF-G: postpartum hepatitis flare group; NPHF-G: no postpartum hepatitis flare group.

**Table 5:** Risk factors of postpartum hepatitis flare.

Factors	*β*	Standard error	Wald	*P*	OR	Incidence risk ratio (95% CI)
Anti-HBV therapy	−1.029	0.267	14.835	≤0.001	0.357	0.212-0.603
TBIL (intrapartum)	−0.173	0.055	9.890	0.002	0.841	0.755-0.937
HBcAb (intrapartum)	0.195	0.049	15.561	≤0.001	1.213	1.103-1.339
ALT (pregnancy 32nd week)	0.065	0.015	18.099	≤0.001	1.067	1.036-1.099

ALT: alanine aminotransferase; HBcAb: hepatitis B core antibody; HBV: TBil: total bilirubin.

## Data Availability

The datasets used and/or analyzed during the current study are available from the corresponding author on reasonable request.

## Abbreviations

ALT: Alanine aminotransferase
AST: Aspartate aminotransferase
TBil: Total bilirubin
DBIL: Direct bilirubin
HBeAg: Hepatitis B e antigen
HBsAg: Hepatitis B surface antigen
HBV: Hepatitis B virus
HBV DNA: Hepatitis B deoxyribonucleic acid
SD: Standard deviation
ULN: Upper limit of normal
WBC: White blood cell
PLT: Platelet
HGB: Hemoglobin
ALB: Albumin
PHF-G: Postpartum hepatitis flare group
NPHF-G: No postpartum hepatitis flare group
MTCT: Mother-to-child transmission
T-G: Anti-HBV therapy group
C-G: Control group (anti-HBV therapy group).
